# Internet False News Information Feature Extraction and Screening Based on 5G Internet of Things Combined with Passive RFID

**DOI:** 10.1155/2021/9696472

**Published:** 2021-12-30

**Authors:** Dahai Hu, Qiong Xia

**Affiliations:** School of Journalism and Communication, Wuhan University, Wuhan 430072, China

## Abstract

In this paper, the authenticity of news information on the 5G Internet of Things (IoT) is studied, and a network false news information screening platform is designed and optimized by IoT combined with passive RFID. The electronic license chain based on data sovereignty is established, in which, combined with the identity identification and strong correlation ability based on the electronic license chain, a cross-industry, cross-business, and cross-field behavior record base database is formed; then, a digital library is constructed based on this base library; finally, through data sharing and management, a false news information feature extraction and screening platform is formed for the orderly management and reasonable dispatch of government resources and reducing various risks. The main functional modules implemented by the platform are the acquisition of news data and comment data, the retrieval and analysis of news data, the false detection of online news, and the visualization of false news data. However, there is still much public who are not aware or do not understand that news truth is this dynamic form. Therefore, this paper aims to inform the public that news truth in news context is a dynamic process by 5G Internet of Things combined with passive RFID. The public understands the circumstances where news truth may be dynamic truth to avoid being misled by false news.

## 1. Introduction

News truth is the lifeline of news; the news, true or not, will affect the public's trust in news; therefore, the press always takes truth as the life of news and insists on news truth as one of the most basic business norms and the most important working principles [1]. Scholars in different periods will continue to change the research and results of news truth with the requirements of technology and society, constantly exploring and deepening that the connotation of news truth is the source of making news alive and everlasting. In recent years, news inaccuracies have frequently appeared, mostly in new media platforms, and the status and authority of news media have been greatly impacted, and the truthfulness of news has been questioned, so in this context, it is of practical significance to rethink the truthfulness of news reports in the context of news [2]. By reexamining the dynamic process of news authenticity, journalists, especially the audience, can understand that news authenticity is more prominent in the new media context as a dynamic expression and realize that “news authenticity is a dynamic process” to reach a consensus and reshape the authority of news media, which is important to reduce false news and maintain social stability. And it is of great significance to reduce false news and maintain social stability [3].

In the network news release link, the media plays an important role, and creating a healthy network environment requires the media to supervise each checkpoint. Traditional media is strengthening integration and development, continuing to play the role of authoritative media in the Internet environment, using the Internet to present news content in traditional media to users in more diverse forms, but for now, traditional media has formed in the Internet of Things [4]. The influence of Internet media is growing. Therefore, the governance of Internet false news incidents still needs to rely on Internet media, by improving the media literacy of online media and exploring the characteristics of its gate-keeping mechanism, effectively preventing the spread of online false news incidents [5]. News production in news contexts affects the production logic of news truth; news verification before reporting is converted to verification after reporting, and news truth is transformed from conclusion truth to process truth, all of which are closely linked to the characteristics of news contexts. The algorithmic mechanism is a new thing in the Internet era, and the research in this field in the academic industry is not yet mature. As the core mechanism of Internet information flow, machine algorithms have a certain impact on citizens and society through the collection and processing of information distribution [6]. The balance between technical rationality and value rationality can make technology better serve human beings, and the opposite is easy, to put the cart before the horse. How to balance the two requires contemporary researchers to propose more advanced and contemporary theories as to the basis. Most scholars have selected a definite ethical issue to study the phenomenon of this new phenomenon, but few scholars have looked at the essence of the phenomenon to analyze its intrinsic problems.

Network fake news is defined as false information posted by users on social media, that is, news information or rumors that are not consistent with the facts and cause a certain amount of public opinion released by individuals without official confirmation. Chapter 1: Introduction: this chapter first summarizes the research background and significance, research content, development trend, and application fields of Internet false news information feature extraction and screening based on 5G Internet of Things combined with passive RFID and finally gives a detailed description of the main research content of this article and the organization structure of the article. Chapter 2: Research on the Internet of Things News Screening Platform: the current research status is introduced. At the same time, an algorithm for feature extraction and screening of Internet false news information based on 5G Internet of Things combined with passive RFID is proposed, and an optimization platform for Internet false news information is established. Chapter 3: Result Analysis: with the optimization algorithm proposed in this paper as the core, the experimental process and experimental results are described and analyzed, and the effectiveness of the method proposed in this paper is verified through comparative experiments. Chapter 4: Conclusion: this chapter summarizes the full text, summarizes the main points of the full text, and looks forward to future work.

## 2. Research on 5G IoT News Feature Extraction Platform

### 2.1. Related Work

A study by Miloslavskaya pointed out that secure, well-attributed data sources are critical to data accountability, forensics, and privacy [7]. A decentralized trusted cloud data source architecture using IoT is proposed. IoT-based data sources provide tamper-proof records, increase the transparency of data accountability in the cloud, and contribute to the privacy and availability of source data [8]. In the paper, ProvChain is designed and implemented to collect and verify the architecture of cloud data sources by embedding source data into IoT transactions utilizing cloud storage scenarios and selecting cloud files as data units to detect user actions to collect source data [9]. The results of the performance evaluation of this approach show that the source user privacy and reliability of cloud storage applications are minimal, so the source data collection, source data storage, and source data verification are needed [10]. The study by Hoang points out that data-based encryption, especially attribute-based encryption based on ciphertext policy, plays an important role in data sharing [11]. The study of an efficient and privacy-preserving traceable attribute-based encryption scheme for IoT is proposed. The scheme uses a preencryption technique to quickly generate ciphertexts and hides the attributes of anonymous access control structures by using attribute bloom filters. The source of misused keys can be audited in case of misuse.

Uslu et al. collected official rumor information on news platforms as an experimental data set. Through research, they found that the geographic location and terminal equipment used by users when posting Weibo have an important impact on rumor recognition. The feature is added to the feature set of the rumor, and the rumor detection based on the Weibo platform is realized by constructing an SVM classifier [12]. Kumar combined 5G IoT electronic data to become common evidence, from the perspective of judges reviewing the authenticity of electronic data, explored the possibility of electronic data being tampered within various aspects of collection, extraction, preservation, and transmission due to its intangibility and vulnerability to destruction, as well as the difficulty of discerning the authenticity and integrity of electronic data, which affects the admissibility and probative value of electronic data, and concluded IoT-based technology for multiparty deposition, to ensure the authenticity, security, and validity of electronic data conclusion [13]. Research on the compatibility of UHF RFID and cellular networks is based on reflection modulation and proposes a design scheme for passive cellular IoT systems, including cellular IoT base stations, passive terminal software and hardware architectures, and mainstream benefits compatibility. Although it is still a theoretical study, it can be seen that the research of cellular networks supporting passive IoT has also been put on the agenda, and the research direction of 5G supporting passive IoT access also has a certain foundation. In the past development process of the Internet of Things, the passive Internet of Things seems to have no intersection with the cellular network. Today, the vision of allowing 5G to carry hundreds of billions of Internet of Things access is indispensable for passive IoT support. Driven by this goal, cellular mobile communication networks are closely integrated with passive IoT for the first time and become the future largest group in 5G connections.

Fake news refers to news reports that do not reflect the objective truth and contain false elements and can be divided into two categories: one is news reports in which the communicator intentionally fabricates facts out of thin air for some purpose and disseminates them; the other is news reports that are generally true, but some details of the description appear to be false or intentionally or unintentionally misinterpreted or falsified. Reverse news is “news that is initially reported in the opposite direction, and as the news report goes deeper and deeper, the truth is presented to the readers more objectively and comprehensively, and the readers' position is sharply reversed and they show the opposite attitude from before.” Reversal news is distinct from fake news. This article combines news text similarity features, news and comment data emotional tendency features with some statistical-based user features to construct feature vectors, and uses IoT classifiers to train the data to obtain the final fake news detection model through the model “detect news data and display the classification results in the system.”

### 2.2. Information Feature Extraction Algorithm

In intelligent algorithmic backend applications, the algorithm decides what content can enter the distribution channels, what information each user likes to read, and what news reports can occupy the main part of the distribution content and seem to evolve into the decision of the audience, which will lead to algorithmic news catering to the entertainment needs of the audience, ignoring the impact of the news itself on the public, industry, and society. Usually, post-truth news is the result of a significantly different public opinion sentiment that accompanies modern public opinion and is an important sign of the reversal of public opinion [14]. Fake news will not necessarily be clarified. The “reversal” of reversal news is the process by which the truth is continuously discovered. Reversal news will generally cause strong repercussions and create a strong public opinion situation.

Robots for data collection have become an important source of information for new media; a few days ago, the algorithm recommended news mainly relying on three production push mechanisms: one is the user portrait algorithm, in full accordance with the user hobby mapping recommended information, using the similarity of two or more user attributes to find the same cluster of users. These three content distribution models have in common the pushing model of giving different weights to algorithms to seek attention to the news, which makes it difficult for the public to scientifically select the social and cultural values embedded in the news, which requires gatekeepers to adhere to the confirmation and review of information, to guide the public to rational behavior, and to ensure that objective and accurate news will not be lost in the ocean of information. Therefore, in the stage of intelligent media, the existence of gatekeepers is reasonable, and the breakthrough can be made by personalized news, with algorithms and professional editors acting as gatekeepers, avoiding algorithms occupying the main position of gatekeepers, ensuring that news content meets the ethical and moral requirements of journalism, and reshaping the authority of gatekeepers, as shown in Figure 1.

The news media has the function of guiding social opinion and simultaneously setting important events in society as fixed issues. Although robots have changed the news production and content distribution mode, robots cannot replace the monitoring function [15]. The mass media in the traditional sense represents the public opinion and is a collection of public opinions and issues. Public opinion supervision is completely different from rigid forms of supervision such as administrative supervision; it is a special form of soft supervision without strict regulations and requirements, and thus not compulsory, but it can play a role in educating and spreading mainstream values to the public. The media assumes the role of a public issue person in public opinion supervision, and as robotic writing becomes an important development trend in the media industry, it does not completely change the status of machine algorithms replacing human beings as the main body of supervision, which seems to be a cause for celebration. By continuously adding or deleting features, the accuracy of the model is tested on the verification set to find the optimal feature subset. The wrapped method usually has higher accuracy because of the direct participation of the model, but because each feature changes, the model must be retrained, so the calculation cost is high. Another disadvantage is that it is easy to overfat.

(1) $$\begin{array}{c} F\left(D_{i}\right)\leq H_{i}-\left\|T_{i}\right\|{\left\|\nabla TX\right\|}_{i}\left\|d_{i}N_{i}^{2}\right\|. \end{array}$$

In the digital world, everyone has a physical presence, and all communication and collaboration will be based on the digital world as the norm and core, while the customary physical world becomes an aid and supplement to the digital world. This process is not only the realization of technology. The IoT security gateway reports news information recognizes news information in the unified management platform, and displays news distribution and true and false status in real time. Combined with the internal network isolation and baseline detection of the Internet of Things gateway, it blocks terminal intrusion detection and propagation.

(2) $$\begin{array}{c} X=\underset{N⟶\infty }{\lim}\sum_{i=1}^{N}\beta_{i}^{n}\left(d_{i}-1\right). \end{array}$$

We can achieve objective, fair, and scientific supervision and full supervision of credit evaluation through the comprehensive application of IoT and other technologies and, at the same time, strengthen the supervision of credit evaluation agencies to ensure that their evaluation is fair and untamable [16]. One is to use data sovereignty IoT technology to guarantee the operation right and basic bookkeeping right of IoT, and the core institution of data sovereignty to carry out the support and application of operation, to effectively guarantee the safety of people and national information property; the second is to use IoT technology to supervise the operation process of power operation, livelihood application, public service, and other affairs in the whole process.

To observe *X*, the signal *X* is projected using a matrix of *M* to obtain the observation vector *Y*.

(3) $$\begin{array}{c} Y=A_{i}^{CS}\left(\beta -1\right)\beta_{i}^{n}. \end{array}$$

IoT technologies are devoted to developing key technologies at the protocol and infrastructure layers that can take credit scoring-related data collaboration to a higher level. Meanwhile, a high-performance and secure credit data exchange network based on IoT technology can improve data quality, reduce data collection costs, expand data coverage, and ultimately create better credit scoring models through artificial intelligence used to update and calculate the network parameters that affect the model training and model output to approximate or reach the optimal value, thereby minimizing (or maximizing) the loss function. Therefore, IoT technology can not only play the advantages of high security and benefit-sharing, but also achieve the performance requirements needed for industry scenarios. Formula (4) is a performance statistical function, where *β* represents the statistical type, and *n* represents the statistical period.

(4) $$\begin{array}{c} \beta =\arg\max{\left\|\beta_{i}^{n}\right\|}^{2}. \end{array}$$

Because laws and regulations can only be remedied after the fact through state intervention, while technical rules can be prevented beforehand through code. The function and role of law and code under the Internet society can be considered high and low. However, the translation of legal rules into technical rules is not an easy task. A legal code is a general rule that is essentially ambiguous and written in language; a technical code, in contrast to a legal code, can only be expressed through the code and necessarily relies on algorithmic forms and digital models. While code increasingly mimics or even replaces some of the traditional functions of law in the digital world, in the last few years, especially since the emergence of IoT technologies and smart contracts, the law has also come to display some of the characteristics of code. The feature extraction and screening of false news information are shown in formula (5), where U represents the feature set, *t* represents the collection time, *s* represents the screening method, and *c* represents the extraction method.

(5) $$\begin{array}{c} U_{t}=\frac{y_{i}^{2}\left(t,s\right)\left(1+e^{x_{m}c_{m}\nabla A}\right)}{e^{x_{m}c_{m}\nabla A}}. \end{array}$$

This information recommendation method helps users find the information they are interested in and read daily in a sea of information, reducing the time spent on information search, and people seem to have used to this way of receiving the news [17, 18]. The algorithm replaces the user's way to find information and invariably replaces the individual user's information selection, creating private customization of the information content platform, allowing irrelevant news to be lost in the sea of information, and making the user refuse to receive social issues from other public areas, which will generally reduce the public's social cognitive ability in the long run.

### 2.3. Fake News Optimization Combined with Passive RFID

It is reflected in the internal verification process of journalists, which is the most reflective link of the main position of journalists and belongs to the prereporting verification. For a long time, journalism at home and abroad has always held “news truth” as the lifeline of news and requires journalists in the process of news reporting must ensure that news events are reported in a completely true and objective way; therefore, journalists in the acquisition of newsworthy information about recent events must go through a verification [19]. In the process of verification, journalists must collect as many accounts as possible from different parties or eyewitnesses to restore and reproduce the actual event from multiple angles and in a comprehensive manner. Verification of news content is a necessary process to ensure that news reports are authentic and credible, and so is news production.  Figure 2 represents the optimized architecture of the news information screening platform combined with passive RFID. The main purpose of the online fake news detection system is to detect online fake news. The system contains four main functional modules, namely, the acquisition module of Internet of Things network news data and comment data, the analysis and retrieval module of network news data, and the network false news detection module, and the data analysis result visualization module, among which the IoT false news detection module is the most important functional module in the system.

The process of authenticity identification service design is as follows: firstly, the client node in the IoT platform calculates the digital digest of the local file, calls the authenticity identification API, and initiates a request to the server node; then the server node authenticates the network certificate held by the node, and if the verification passes, the node is authenticated, and the file access authority is verified; if the verification fails, an error message is returned, and the call is terminated [20]. If the verification passes, and the nodes on the chain reach consensus, the relevant data in the process will be written to the block and packaged, and the corresponding message will be returned to the client node; otherwise, an error message will be returned, and the call will be terminated, thus ending the authenticity identification service.

News reporting is the reporting of newly occurring or newly discovered facts, and the object of its reporting is the matter that is available in the objective world. Epistemology believes that the objective material world is always in the process of movement and change; therefore, from the perspective of the object to explore the dynamic process of news reality, it is necessary to clarify a point of view; that is, the fact itself is in a state of motion of constant change and development, and then the news reality corresponding to the event will also necessarily be in a dynamic process [21]. Many news reports of the event with special characteristics and complexity, in those instant reports of the news process, due to the reporting of the event at the time of some matters or details have not been fully revealed; instant reporting can only present the facts that have been revealed partly, and then with the development of the event for follow-up reports, in such a continuous and dynamic reporting, the overall reality of the news event also shows a dynamic presentation. In such continuous and dynamic reporting, the overall truth of the news event is dynamically presented. Second, the fragmented news text in the news context can hardly present the complicated and objective world completely. Therefore, the news truth from the object perspective is also in a dynamic development process with the development of news events.

Traditional mainstream media are limited by technology to a longer time limit for news reports and limited channel resources, and news reports are more inclined to one-time final reports, with many news being reported only after the development of the matter is over, and after in-depth digging and verification by reporters. Therefore, the content of these reports is completed, and the news reality shown to the audience is also more complete. Only a small number of news events with a relatively large impact, such as sudden disaster events, are released for the first time to inform the public, and then follow-up reports of the events are released continuously. In contrast, news reporting in the news communication context has shown recent changes and forms due to the real-time nature of news releases and the brevity of news content, as well as the competitive pressure of information release channels. To grab headlines, professional news media often release concise news stories to let audiences know that something has happened before it is finished and then follow up on the news to grab headlines. The complex communication ecology of the news communication context drives news reports to keep pace with the development of news events and makes the dynamic characteristics of news truth more prominent. In the news communication context, news truth also presents a gradual and dynamic process because of the development process of news events.

IoT technology has the characteristic of “data sharing,” which refers to the sharing of data storage and exchange level [22–25]. The IoT network makes multiple copies of the data on the chain and stores them on multiple storage nodes at the same time, so from the data point of view, the data is shared to multiple nodes and can be downloaded from any node. However, from the perspective of data content, the platform can encrypt the data content through encryption technology. Even if we get the encrypted data, we cannot access the actual information contained in the data without the decryption key. Therefore, the platform identifies the legitimate users based on the account mechanism, assigns the users the contents they have a right to view and the decryption key through the permission mechanism, and ensures data security by encrypting the data on the chain through the encryption technology. The platform supports the information security mechanism based on permission and encryption functions. In simple terms, the integrity file platform needs to be completed with a system that supports identity-based permission control and password mechanism and only responds to user requests through the IoT gateway, specifically including filtering out requests from illegal users and cross-authority requests from legitimate users.

All data compiled in this study included all online news headlines from seven major websites with names in the title and time from 2010 to 2019. A total of 8825000 news headlines were collected, and the results are shown in Table 1.

The network false news detection module detects false news based on the constructed test model. In the system design of this article, the test model generated in advance based on the training data is stored in a txt file, and the news collected in this system can be detected and identified. When you click on fake news analysis, you can use a visual mode to show the trend changes in the number of comments related to the news and the analysis results of the text and comments.

## 3. Analysis of Results

### 3.1. News Information Feature Extraction Results

Social platforms such as microblogs, which are based on Internet technology, have the functions of both information dissemination and social interaction, allowing users to express their opinions or respond to others' opinions through comments, retweets, and private messages. The dissemination of information on the microblogging platform is not restricted by time and space, and users can spontaneously and actively participate in discussions, actively verify the information, and provide other information after news reports are released, which invariably constitutes a unique “self-clarification” mechanism in the online environment, as shown in Figure 3. Among them, the information of the day accounted for the highest proportion, reaching 32.5%, and the proportion of information over two weeks was the lowest, accounting for only 11.2%.

Among them, the information of the day accounted for the highest proportion, reaching 32.5%, and the proportion of information over two weeks was the lowest, accounting for only 11.2%. Those that are longer than two weeks are the event itself that is still in the development process, so it takes a relatively long time. Overall, the real clarification time of news in the context of Weibo is relatively short, and clarification can be obtained relatively quickly.

Filter out the useless comment data, and extract the features of Weibo content and comment-related content, based on the original feature, the combination of the original feature and the newly extracted text feature, and the original feature and the newly extracted text feature. The combination of text and comment features was experimented separately. Through the data in the test, the reliability and performance stability of the IoT platform are reported. However, in the process of false analysis of news and sentiment analysis, due to the processing of more data, there will occasionally be longer response times. The detection efficiency of the IoT platform still needs to be improved.

Through the analysis of 60 cases and overall, it is found that 73.33% of the news reports present dynamic reality because of the lack of verification or being reported and reprinted without verification, 11.67% of the news reports are fictitious news to win the audience's attention, and other factors include poor professionalism of journalists, unfinished events, and lack of authoritative information, as shown in Figure 4.

Figure 4 reveals that the main reason for the prominence of the dynamic process of news in the current microblogging context lies in the lack of prerelease verification of news reports. The cause for the widespread of many fake news stories is that professional news media simply copy and paste them without verifying the news content, all at the cost of losing the credibility and authority of the news. The phenomenon of backstage news foregrounding has emerged along with the weakening of the verification process in the professional news media. Goffman introduced theatrical elements and staging techniques into interpersonal interactions and put forward “drama theory,” which compares interpersonal interactions to personal performances and proposes the concepts of front stage and backstage. The front stage performance is more formal, while the backstage performance is relatively relaxed and unruly. Some studies have introduced Goffman's drama theory into the news reporting industry and explored the relationship between news media and audiences, arguing that news also has a front and backstage, in which the production work before the release of news reports is the backstage, TV, newspapers, and official microblogs belong to the front stage, and each news report is treated as a front stage performance, and the news reports that audiences are exposed to are front stage acts, and the previous news front and backstage boundaries and behavioral segmentation. The previous news front and backstage boundaries and behaviors are relatively clear. However, in the microblogging context, the front and backstage boundaries of news reports are blurred, because the verification process of news media is weakened, which reduces the authenticity of news reports, and many news are reported after netizens raise questions, or some knowledgeable people point out that the news reports are not in line with the actual situation, which leads to the verification behavior of the backstage being moved to the front stage and the front stage turning into the backstage. This is one of the reasons why news reality in the microblogging context presents a dynamic process.

Figure 5 shows the changing pattern of network size at each dissemination stage, and the numbers of nodes and edges of the network are the indicators of network size. Among the four stages of online opinion dissemination, the numbers of nodes and edges are the largest in the outbreak period with 3864 and 1610, respectively, indicating that the network scale is the largest at this time, and most microblog users are involved in opinion dissemination. In the latent stage, the network size is the smallest, and the numbers of nodes and edges are small, but the difference is not very large, while, in the growth and decay stages, the number of nodes of the network is greater than 1000, and the number of edges is about 330, indicating that although many users participate in the discussion in these two stages, only a small number of users have retweeting relationships with each other.

From the trend of the maximum node degree of network nodes in Figure 5, it can also be seen that although the maximum node degree of network nodes differs significantly from the network nodes and edges in terms of number, the trend of change does approximate the same. The maximum node degree of network nodes also reaches its maximum value during the outbreak of public opinion. News from different information sources is brought together, and news truth becomes more complex and difficult to discern. Often, the public must increase their capacity to select and screen information and consciously develop their thinking about news counterfeiting. Do not jump to conclusions blindly, but keep a skeptical attitude. If necessary, you should combine life experience and common sense to make judgments, just like in daily life, and not believe in things that fall from the sky; similarly, in the microblogging platform, you should not believe in information that is inconsistent in wording and things that do not make sense and also be easily convinced and spread it, but you should reserve your opinion about some uncertain information. It is better to wait patiently for the professional media to provide authoritative information, to minimize the negative impact brought by the process of real news dynamics.

### 3.2. Platform Optimization Results

As shown in Figure 6, the latent period of public opinion has both large network density and average network degree, but the average shortest distance length of the network in this period is particularly large, which makes the connection between users in the latent period very close but hinders the dissemination of public opinion information more difficult due to the longer dissemination path. While the values of network density in both the outbreak and decay periods of public opinion are relatively small, and information transmission is not very easy, the average shortest distance length of the network is much smaller than the rest of H periods, and the average degree of the network is also relatively large, so that, in the outbreak period, public opinion information is transmitted quickly among users, and communication among users is more frequent; on the contrary, in the decay period, the average shortest distance of the network is very large, and the average degree of the network is relatively small, so that, in the decay period, public opinion information is spread slowly, and users are less connected to each other and interact less.

Figure 7 shows the statistics of the number of news retweets. These users have a common characteristic; that is, they have a certain status of speech in the society, and the blog posts and opinions they publish will be responded to by a group of a not small number of people and exert a large influence, which is what we call opinion leaders. These users have a huge circle of fans and a large influence, so they do not have to deliberately publish numerous blog posts or follow others on purpose. When public opinion occurs, the information released by each person only represents the opinion, and the quality of information from certified users is relatively much higher, which also plays a role in the supervision of online information. These users will post or forward blog posts that can represent their emotional tendencies, thus influencing the remarks and emotions of other information recipients and playing a role in the spread of public opinion.

Figure 8 indicates the statistical information of the system node data. The system performance and system operation data of all aspects of the constructed integrity file platform meet the technical requirements, realize the electronic license chain based on data sovereignty IoT technology, and can realize the efficient application of electronic license in anticounterfeiting, impersonation verification, privacy protection, safe sharing, visualization, and authority. This set of integrity file systems built based on integrity data sources with communal sharing in the whole field has laid a solid foundation for the subsequent in-depth research of data sovereignty IoT technology.

In the process of modern news dissemination, the report form of any piece of news has to go through many processing processes. In these processing processes, news facts are recognized, formed into images, latent processing, written expressions, value judgments, and disclosures. There are many links such as publication, and each link is operated by humans. This not only helps ensure the authenticity of the news, but also greatly helps the news writing process and enrichment of the content. It is also the basis for writing good articles. As journalists in an era of unprecedented fierce competition, we should remember that any report we make must be personally and meticulously investigated and researched before it can be published responsibly to a broad audience. As long as this is achieved, the authenticity of the news will be fundamentally guaranteed, and the lifeline of the news media will be fundamentally ensured.

## 4. Conclusion

The paper elaborates the theoretical system, principle, and development process of the key technology of the news information feature extraction platform based on data sovereign 5G Internet of Things and demonstrates and tests the prototype system of the news information screening platform combined with passive RFID. The truth of news reports is as a small part reflecting the overall social reality, and the facts of news reports from different angles and positions that finally present the real picture of the whole society through the stage and dynamic reports. Also, because the production process was more rigorous and thorough during the traditional media era, the truthfulness of the news was better assured. The limited human knowledge of technology and self-knowledge, coupled with the public's blind pursuit of the excitement and novelty of new technologies and the lack of corresponding rational thinking, has exacerbated the degree of ethical misconduct in journalism on some levels. Data sources can be expanded in future research. How to obtain these data from the media and how to analyze fake news purely from a textual perspective are a long-term and meaningful thing, so the screening of fake news still needs to be further investigated. The experiment and analysis of data mining technology are used to identify fake news and thus develop a more accurate fake news screening system.

## Figures and Tables

**Figure 1:** IoT information screening model architecture.

**Figure 2:** Optimized architecture of news information screening combined with passive RFID.

**Figure 3:** Length of news true clarification.

**Figure 4:** Reasons for news misrepresentation.

**Figure 5:** Network node degree during the decay.

**Figure 6:** Trends in network characteristics at each dissemination stage.

**Figure 7:** Distribution of the number of forwarding.

**Figure 8:** Node data.

**Table 1:** Results of the collected news volume.

Year	Value
2010	779854
2011	805974
2012	1685748
2013	1694715
2014	1005895
2015	1234874
2016	1654287
2017	1029574
2018	900125
2019	958426

## Data Availability

The data used to support the findings of this study are available from the corresponding author upon request.
